RETRACTED

# Tracking of Gymnast's Limb Movement Trajectory Based on MEMS Inertial Sensor

**DOI:** 10.1155/2022/5292454

**Published:** 2022-04-27

**Authors:** Peng Li, Jihe Zhou

**Affiliations:** ^1^College of Physical Education and Health, Zunyi Medical University, Zunyi, 563000 Guizhou, China; ^2^College of Sports Medicine and Health, Chengdu Sports University, Chengdu, 610041 Sichuan, China

## Abstract

In order to track the limb movement trajectory of gymnasts, a method based on MEMS inertial sensor is proposed. The system mainly collects the acceleration and angular velocity data of 11 positions during gymnastics by constructing sensor network. Based on the two kinds of preprocessed data, the parameters such as sample mean, standard deviation, information entropy, and mean square error are calculated as classification features, the support vector machine (SVM) classification model is established, and the movements of six kinds of gymnastics are effectively recognized. The experimental results show that when the human body is doing gymnastics, the measured three-axis acceleration values are between -0.5 g~2.2 g, -1 g~2.8 g, and -1.8 g~1 g, respectively, and the static error range accounts for only 1.6%~2% of the actual measured data range. Therefore, it is considered that such static error has little effect on the accuracy of data feature extraction and action recognition, which can be ignored. It is proved that MEMS inertial sensor can effectively track the movement trajectory of gymnasts' limbs.

## 1. Introduction

Human motion capture system is widely used in remote sensing control, athlete training, film production, disease diagnosis, and other fields. Among these application fields, biomedical related fields are one of the most promising and developing fields. Especially in China, after the baby boom in the 1960s and 1970s, these “babies” have gradually reached the retirement age, and the aging of China's population is becoming more and more serious [1]. As people grow older, especially after the age of 50, they face this mental and physical health challenge. Health problem is one of the most important factors affecting the quality of life. With the gradual improvement of social living standards, people pay more and more attention to health problems. Some health problems, such as arthritis, stroke, and Parkinson's disease, have one thing in common, which has a great impact on the elderly's ability to exercise and move. In order to understand, control, and prevent these diseases, it is very necessary to track, collect, and analyze the patient's behavior. Without affecting the patient's normal life, the patient can wear wearable sensing devices to monitor the patient's physical condition in real time, so that the medical staff can better understand the patient's condition, so as to provide a more accurate basis for the diagnosis and treatment of diseases [2]. Motion capture system is widely used in inertial navigation, virtual reality, biomedicine, man-machine control, sports, and other fields. As shown in Figure 1, it has attracted more and more attention. Continuous monitoring of patient information provided by motion capture equipment is very important to find their health problems in time. In addition, the movement behavior and position of elderly patients can also be tracked in real time, so that they can be treated in time in case of emergency. A motion capture system may include various types of wearable sensor devices, such as sensors monitoring the physiological characteristics of patients, such as mobile current scanners, and motion characteristics, such as accelerometers, gyroscopes, and magnetic flux sensors. These sensors can monitor the patient's health status and limb activity information [3]. Wireless wearable inertial sensing device allows to estimate the unrestricted rapid movement of limbs, which can significantly improve the performance of motion capture, and it is convenient and free. Motion tracking is also acceptable in daily life. Combined with wireless sensor network technology and MEMS technology, a human motion capture system is developed, and the trajectory tracking algorithm is improved. The human motion capture system can measure the motion direction and angle of human joints. The pose information of important joint points of human body collected by micro inertial sensor is sent to PC through wireless sensor network, and the server on PC receives it, so as to drive the human model on PC and realize the real-time simulation and simulation of human motion. In recent years, outdoor tracking and navigation systems have been widely used and developed, such as global positioning system (GPS) and triangulation, which can provide accurate geographic and absolute location information. Due to the blocking of signal by buildings, GPS indoor positioning is unreliable, which has a large error. By combining GPS and inertial sensor, better results are obtained than GPS in collecting position information. The interference received by GPS in indoor positioning is uncertain. In this paper, only inertial sensors are used for trajectory tracking and positioning. The trajectory tracking system is a supplement to the motion capture system. It is planned to combine the two to more accurately realize the real-time capture of human motion in the future [4].

RETRACTED

## 2. Literature Review

Zihajehzadeh et al. use GPS to measure the motion trajectory of the object. Due to the influence of complex environment such as terrain or building shielding, the positioning accuracy of the receiver is very poor or even unable to locate. The use of MEMS sensors for motion trajectory measurement does not require the preinstallation of positioning equipment in the sports field, with low cost and flexible operation [5]. Zihajehzadeh et al. adopt MEMS acceleration sensor, which uses the acceleration integration principle to measure and estimate the motion trajectory. However, the cumulative error of the acceleration sensor is too large, which affects the measurement effect [6]. Copeland et al. propose a recognition method to extract the information features of MEMS inertial sensor data, that is, to recognize gestures by extracting the feature quantities and variation laws of acceleration and angular velocity. This method cannot recognize gestures related to time sequence, and there are some limitations in the recognition of complex gestures [7]. Tu et al. improve the feature extraction method and added time series to recognize gestures related to time sequence. However, only the acceleration sensor is used, which limits the motion attitude of the equipment and brings inconvenience to the operator [8]. Vysock et al. use distributed sensor networks for human motion recognition and proposed a linear settlement method to process sensor network data, but there are many sensors, large amount of data, and low real-time performance [9]. Sebastijan and Matjaz collect human motion data by using the mobile phone's own accelerometer and gyroscope sensor, analyze the time domain and frequency domain of the original data, and extract the relevant eigenvalues. Then, the recognition results are obtained by using j48 decision-maker combined with Markov model, which can recognize people going upstairs and downstairs, running, walking, stationary, and so on. However, the algorithm can only recognize a certain state of people for a period of time and cannot count actions [10]. Mekruksavanich and Jitpattanakul also use decision tree and windowing to recognize human squatting, lying, and other actions. However, due to windowing, it is still impossible to segment any single action, and it is difficult to realize the counting function [11]. Doddabasappla and Vyas design a hybrid two-dimensional position sensing system and applied it to the mouse. The system measures the hand motion acceleration through MEMS accelerometer and then converts it into two-dimensional position coordinates through quadratic integration algorithm [12]. Wei and Fan propose that using two biaxial acceleration sensors can better measure the angle of the joint under static conditions, but it is difficult to eliminate the inertial acceleration interference of limb movement under dynamic conditions [13]. Lin and Lian use MEMS accelerometer and gyroscope for data fusion, which effectively suppressed the influence of acceleration sensor error on measurement accuracy [14].

RETRACTED

Based on the current research, a method based on MEMS inertial sensor is proposed. The system mainly collects the acceleration and angular velocity data of 11 positions during gymnastics by constructing sensor network. Based on the two kinds of preprocessed data, the parameters such as sample mean, standard deviation, information entropy, and mean square error are calculated as classification features, the support vector machine (SVM) classification model is established, and the movements of six kinds of gymnastics are effectively recognized.

## 3. Gymnastics Movement Recognition System

The hardware part of the gymnastics movement recognition system is mainly composed of motion detection module, main control module, and wireless data communication module, as shown in Figure 2. Among them, the motion detection module is MPU6500 chip, and its performance indexes are shown in Table 1. A three-axis accelerometer and a three-axis gyroscope are integrated in the chip, which are used to collect the acceleration data and angular velocity data of human action, respectively, and realize the data output through three 16 bit ADCs. In order to accurately track fast and slow motion, the measurement ranges of gyroscope and accelerometer are set to be adjustable in the range of ±250°/s to ±2000°/s and ± 2 g to ±16 g, respectively [15].

The main control module is the ARM microcontroller STM32F103ZET6 chip, which is mainly used to receive and process the original data of gymnastics from the motion detection module. The chip has up to 112 I/O ports, 11 timers, and 13 communication interfaces and can connect up to 8 sensor nodes. In addition, this paper selects the ESP8266WiFi module with high-speed transmission function to realize wireless data communication, which can transmit data to PC in real time.

### 3.1. Information Extraction

With the continuous development of mobile electronic devices and sensors such as smart phones, smart phones embedded with MEMS sensors have been widely used in life. Therefore, this paper uses mobile phones as experimental hardware equipment to carry out gesture recognition based on acceleration sensors and gyroscope sensors. The operator holds the mobile phone, and the motion trajectory of the hand is the same as that of the mobile phone, so the motion trajectory of the mobile phone can be obtained. Obtain the data of acceleration sensor and gyroscope sensor in mobile phone through a simple Android application, and send the data to PC in real time. Then, process the data on the PC side.

RETRACTED

#### 3.1.1. Acceleration

Acceleration is done by the MEMS accelerometer in three directions: *x*, *y*, and *z*. The orientation of the accelerometer is defined as follows: the short side of the wire is laid on a table parallel to the body. The direction from the lower right corner to the lower left corner of the cell phone is the *x*-axis direction, the direction from the upper left corner to the lower left corner is the *y*-axis direction, and the direction is perpendicular to the plane is the direction of the *z*-axis. As shown in Figure 3, the CD is a short section of the phone. Acceleration includes gravitational acceleration *g*; i.e., when the cell phone is stationary and horizontal, the acceleration of the *x*- and *y*-axes is theoretically 0, and the acceleration of the *z*-axis is the gravitational acceleration *g*. The acceleration curve is shown in Figure 4. The horizontal axis is time, the unit is s, the vertical axis is acceleration, and the unit is m/s^2^, i.e., the output value of the MEMS acceleration sensor [16].

Assuming that the sampling starts from time *t*_0_, according to the integration principle, the displacement *s*(*t*) in the continuous time domain *t*_0_ − *t* and the instantaneous velocity *v*(*t*) at time *t* are expressed as follows:

(1) $$\begin{array}{c} s\left(t\right)=\int_{t_{0}}^{t}v\left(t\right)dt+s\left(t_{0}\right),\\ v\left(t\right)=\int_{t_{0}}^{t}a\left(t\right)dt+v\left(t_{0}\right). \end{array}$$

The movement displacement of the hand can be obtained by double integration of the obtained acceleration. The PC terminal obtains the motion acceleration of the hand in real time and integrates the accelerations in three directions to obtain the instantaneous velocity and spatial cumulative motion trajectory of the hand.

#### 3.1.2. Angular Velocity

The angular velocity is provided by MEMS gyroscope sensor, which is divided into three axes: *x*, *y* and *z*. During hand movement, the mobile phone may turn over in space. At this time, the coordinate system of the acceleration sensor no longer coincides with the absolute motion spatial coordinate system of hand movement; that is, the gravitational acceleration will cause offset components in the *x*-, *y*-, and *z*-axes of the acceleration sensor. In order to solve this problem, MEMS gyroscope sensor is added [17]. The corresponding relationship between the relative coordinate system and the absolute coordinate system is shown in Figure 5. The solid line is the reference coordinate system, that is, the absolute coordinate system, and the dotted line is the coordinate system where the sensor is located, that is, the relative coordinate system.

RETRACTED

In the process of data acquisition, factors such as unconscious jitter of human body, sensor position offset, or interference between sensors may cause acquisition errors, which may affect the accuracy and accuracy of action recognition. The interference signal in the original data is inevitable, but its influence can be minimized through some technologies and methods, such as sensor correction, normalization, and data filtering.

The experiment uses the mean filtering method to remove most of the interference factors in the original data. As shown in Figure 3, the filtered data curve is smoother and suitable for data feature extraction. In addition, it can be seen from Figure 6 that although the acceleration and angular velocity curves of the three axes have obvious periodic variation laws, the periodicity of the *y*-axis acceleration is more prominent. Therefore, the subsequent analysis and identification are based on the *y*-axis acceleration data [18].

### 3.2. Realization of Spatial Positioning

Since the collected data of MEMS acceleration sensor is discrete, set the sampling time interval of the sensor as Δ*t*, and after iteration,

(2) $$\begin{array}{c} r\left[o\right]=r\left[o-1\right]+\frac{b\left[o\right]+b\left[o+1\right]}{2}\cdot \Delta t\left(o>1\right), \end{array}$$

(3) $$\begin{array}{c} e\left[o\right]=e\left[o-1\right]+r\left[o-1\right]\cdot \Delta t+\frac{1}{4}\left(c\left[o\right]+b\left[o-1\right]\right)\cdot \Delta t\left(o>1\right). \end{array}$$

In formulas (2) and (3), *r*[*o*] is the instantaneous velocity at time *t*_*o*_, *c*[*o*] is the acceleration at time *t*_*o*_, and *e*[*o*] is the cumulative displacement in time period 0 − *t*_*o*_.

The output data of the MEMS acceleration sensor is the acceleration in the *x*, *y*, and *z* directions. The instantaneous velocity of the hand along the *x*-, *y*-, and *z*-axes of the acceleration sensor at time *t*_*o*_ can be calculated according to

(4) $$\begin{array}{c} r_{x}\left[o\right]=r_{x}\left[o-1\right]+\frac{b_{x}\left[o\right]+b_{x}\left[o-1\right]}{2}\cdot \Delta t\;\left(o>1\right),\\ r_{y}\left[o\right]=r_{y}\left[o-1\right]+\frac{b_{y}\left[o\right]+b_{y}\left[o-1\right]}{2}\cdot \Delta t\;\left(o>1\right),\\ r_{z}\left[o\right]=r_{z}\left[o-1\right]+\frac{b_{z}\left[o\right]+b_{z}\left[o-1\right]}{2}\cdot \Delta t\;\left(o>1\right). \end{array}$$

Similarly, the motion displacement of the hand part along the *x*, *y*, and *z* directions of the acceleration sensor at time *t*_*o*_ can be calculated, as shown in

(5) $$\begin{array}{c} e_{x}\left[o\right]=e_{x}\left[o-1\right]+r_{x}\left[o-1\right]\cdot \Delta t+\frac{1}{4}\left(b_{x}\left[o\right]+b_{x}\left[o-1\right]\right)\cdot \Delta t,\\ e_{y}\left[o\right]=e_{y}\left[o-1\right]+r_{y}\left[o-1\right]\cdot \Delta t+\frac{1}{4}\left(b_{y}\left[o\right]+b_{y}\left[o-1\right]\right)\cdot \Delta t,\\ e_{z}\left[o\right]=e_{z}\left[o-1\right]+r_{z}\left[o-1\right]\cdot \Delta t+\frac{1}{4}\left(b_{z}\left[o\right]+b_{z}\left[o-1\right]\right)\cdot \Delta t. \end{array}$$

Then, the spatial position coordinates of the hand at time *t*_*o*_ are(*e*_*x*_[*o*], *e*_*y*_[*o*], *e*_*z*_[*o*]).

RETRACTED

### 3.3. Motion Recognition Algorithm

The basis of action recognition is the classification feature recognition of data samples. The commonly used algorithms include *k*-nearest neighbor (KNN), Naive Bayes (NB), decision tree (CART), and SVM. Among them, SVM algorithm has the characteristics of good generalization, unique global optimal solution, and robustness. It shows unique advantages in solving nonlinear and finite sample classification problems. At present, it has been widely used in various classification and recognition problems. Based on the idea of SVM classification. Based on the motion data collected by multisensor network, the accurate recognition of gymnastics is realized. The process includes two parts: action segmentation and classification recognition. Firstly, the original acceleration and angular velocity data representing gymnastics movements are collected, and the mean filtering method is used to smooth the data to eliminate the spike or sudden change interference in the data. Then, the processed data are segmented and feature extracted. Finally, SVM algorithm is used to train and recognize the model [19].

The key step of motion recognition based on motion acceleration and angular velocity data is to extract parameter features that can distinguish different actions. In this paper, sample mean, information entropy, variance, mean square error, maximum, and minimum are used as parameter features. For multiclass features, SVM classifier is used for action recognition. The accuracy of SVM classifier in gymnastics movement recognition is closely related to the selection and training of classification model. The commonly used models are roughly divided into two types: the general model with strong universality and the diversified model designed for personalized experimenters. In order to ensure the recognition accuracy and simplify the experimental process, a general model with strong universality is adopted in this paper. By precollecting the original data of gymnastics from multiple experimenters, multiple models are constructed and trained. And the best classification model is selected according to the training results. This method does not require multiple experimenters to participate in the experiment at the same time but comprehensively considers the characteristics of different individuals, so it can greatly improve the classification efficiency. For the classification and recognition of gymnastics movements, it is necessary to select a kernel function of SVM to classify and train the sample model. Therefore, selecting the appropriate kernel function is the focus of SVM classification and recognition. At present, the commonly used kernel functions of SVM are linear kernel function, polynomial kernel function, Gaussian kernel function, and so on. In order to obtain higher recognition rate, this paper uses three kinds of kernel functions to recognize body side motion, respectively. The research shows that the recognition rate based on linear kernel function is the highest, reaching more than 97%, which is obviously better than other kernel functions. Therefore, linear kernel function is selected for training to obtain the final classification model. Because gymnastics movement recognition is a multiclassification recognition problem, it is necessary to expand the SVM classifier based on two classification model to multiclassification problem. Here, the one-to-one classification method is used to expand it. Assuming that there are *K*-class samples to be identified in gymnastics, it is necessary to establish *K* (*K* − 1)/2 binary SVM. The classifier is constructed as follows:

(6) $$\begin{array}{c} \begin{array}{c} \min\left\{\frac{1}{2}\left\|w^{2}\right\|+C\overset{ls+lt}{\underset{i-1}{\sum }}\xi_{i}\right\},\\ s\neq t,s,\\ t\in \left\{1,2,\cdots ,N\right\}, \end{array}\\ y_{i}\left(w_{st}\cdot x_{i}+b_{st}\right)\geq 1-\xi_{i}, \end{array}$$

where *C* is the penalty factor and *ξ*_*i*_ is a relaxation variable.

RETRACTED

The basic idea of one-to-one SVM classification is to construct a binary SVM with optimal decision between each two different training samples, transform a multiclassification problem into multiple binary classification problems, and then take out the sample points of class s and class *t* (1 ≤ *s* ≤ *k*, 1 ≤ *t* ≤ *k*, *s* ≠ *t*). The optimal decision function constructed by the binary classification SVM algorithm is

(7) $$\begin{array}{c} f_{st}\left(x\right)=\underset{SV}{\sum }a_{i}^{st}y_{i}K\left(x_{i},x\right)+b_{st}. \end{array}$$

Two different samples are identified by SVM classifier. If the sample belongs to class *s* sample, the voting of class *s* sample is increased by 1. If the sample belongs to class *t* sample, the vote of class *t* sample shall be increased by 1. Finally, the final classification result is the one with the largest number of votes.

## 4. Results and Analysis

### 4.1. Experimental Scheme

In order to verify the accuracy and difference of gymnastics movement recognition, 10 healthy male/female college students were selected to participate in the experiment. The sensor device collects the gymnastic movement data of the experimenter at the sampling frequency of 50 Hz, including six typical gymnastic movements, such as stretching, chest expansion, body side, body rotation, kicking, and whole body. Each experimenter completes the above actions according to his/her own habits, and there is no constraints on the experimenter in the process of data collection.

### 4.2. Results

In order to effectively evaluate the recognition effect of SVM algorithm, four recognition algorithms of KNN, NB, CART, and SVM classifier are used to recognize six kinds of gymnastics. The comparison results of recognition rates are shown in Figure 7. It can be seen that SVM recognition algorithm has a high recognition rate for each gymnastics movement, while other algorithms have a poor recognition rate for one or several gymnastics movements and do not have good universality. Therefore, SVM algorithm is finally selected for recognition in this paper.

Firstly, the three-axis acceleration data is selected as the recognition data of gymnastics, and the SVM classification algorithm is used to recognize six kinds of gymnastics, and the results in Table 2 are obtained. It can be seen from the data in Table 2 that the overall recognition rate of different gymnastics by the method proposed in this paper is different. For the chest enlargement movement, its movements are mainly concentrated in the upper limbs of the human body. The movements at the wrists and arms have large amplitude and many changes. The characteristic value of the movement data is high, and the recognition rate can reach 100%. The range of motion of legs and feet is small, and the positions of hips and waist are easily affected by factors such as sensor sliding, resulting in dislocation of motion recognition, resulting in low recognition rate.

In order to further improve the accuracy of action recognition, this paper extracts the features of three-axis acceleration and angular velocity data and uses SVM algorithm for further recognition. The results are shown in Table 3. Compared with the acceleration data features alone, the actions of legs, feet, hips, and waist can be better recognized based on the three-axis acceleration and angular velocity data features. The recognition rate of each action is more than 97%, and the recognition effect is significantly improved.

RETRACTED

Due to the influence of external environmental temperature, noise, and other factors, the sensor inevitably has inherent drift. Moreover, in the process of gymnastic data acquisition, the rapid and significant changes of human movement will also affect the reliability of sensor wearing. Therefore, there must be some errors in the collected data, which will affect the accuracy of feature recognition and action recognition rate. In order to accurately evaluate the influence of sensor inherent error on action recognition, the acquisition range of MPU6500 acceleration sensor is set to ±16 g (corresponding sensitivity is 2048 LSB/g). The following steps are used to measure the static error of the sensor.

Place the MPU6500 sensor horizontally on the desktop to make it in a resting state. First, make the plane formed by its *x*- and *y*-axes parallel to the desktop, then the *z*-axis is perpendicular to the desktop, and the specified positive direction is up. Theoretically, the sensor system at this time is only affected by gravity, so the acceleration in *x*- and *y*-axes is all 0 g, and the acceleration in *z*-axis-positive direction is 1 g. The difference between the actually measured three-axis acceleration data and the ideal value is the static error of the sensor. Similarly, when the positive direction of *x*- and *y*-axes is perpendicular to the desktop upward, it can be obtained that the acceleration in the positive direction (+*X*, +*Y*) of *x*- and *y*-axes are is 1 g, the acceleration in the negative direction (−*X*, −*Y*) is -1 g, and the acceleration in other directions is 0 g.

Under the above experimental conditions, the static acceleration errors of each axis of MPU6500 sensor are measured, respectively. The results are shown in Table 4. It can be seen that under various axial settings, the error range of three-axis static acceleration is limited to ±0.03 g and will not change with the axial change. When the human body is doing gymnastics, the measured three-axis acceleration values are between -0.5 g~2.2 g, -1 g~2.8 g, and -1.8 g~1 g, respectively. Compared with this, the static error range accounts for only 1.6%~2% of the actual measurement data range. Therefore, it is considered that such static error has little impact on the accuracy of data feature extraction and action recognition and can be ignored. At the same time, it can also be seen from the data in Table 4 that when multiple sensors are at rest at different positions of the human body, the axial height of each sensor is unified. After gymnastics, the axial direction of each part will inevitably change randomly, but this does not affect the static error range of each axial direction of the sensor. Therefore, it shows that when the human body is in motion, the inherent error of the sensor will not affect the recognition effect of gymnastics.

RETRACTED

## 5. Conclusion

The gymnastics movement recognition system based on multi-MEMS sensor fusion designed in this paper can effectively record the acceleration and angular velocity data of each main joint point of human body in the process of gymnastics, extract the sample mean, standard deviation, information entropy, and other parameters of the two kinds of data as the classification features of SVM classifier, and train the classification and recognition model. The results show that the average recognition rate of the sensor system for six gymnastics movements, such as stretching, chest expansion, kicking, body side, body rotation, and whole body, can reach more than 97%. The system and method proposed in this paper can also be used for the action recognition of dance, yoga, martial arts, Tai Chi, and other sports, which will be of great significance to the scientific guidance and systematic training of sports.

## Figures and Tables

**Figure 1:** Application scenario of motion capture system.

**Figure 2:** System hardware structure.

**Figure 3:** Direction of mobile phone sensor.

**Figure 4:** Acceleration curve.

**Figure 5:** Correspondence between relative coordinate system and absolute coordinate system.

**Figure 6:** Waveform comparison of three-axis acceleration and angular velocity data.

**Figure 7:** Recognition results of different classification algorithms.

**Table 1:** MPU6500 sensor parameter settings.

Category	Accelerometer	Gyroscope
Direction	3 axes	3 axes
Measuring range	±16 g	±2000°/s
Power waste	3.2 mA	450 *μ*A
Temperature (°C)	-40~ 85	-40~ 85
Communication mode	I^2^C	I^2^C

**Table 2:** Recognition rate based on three-axis acceleration.

Category	Stretch	Chest enlargement	Whole body	Leg kick	Body side	Body rotation
Single hand	99.46	99.00	100.00	100.00	99.00	97.50
Single arm	99.46	100.00	100.00	95.95	100.00	89.50
Single hip	98.46	94.74	99.00	90.00	96.88	87.42
Waist	99.46	86.84	100.00	82.00	100.00	80.00
Single leg	96.14	92.11	100.00	95.56	100.00	85.00
Single foot	95.14	86.84	100.00	82.50	96.88	87.00

**Table 3:** Recognition rate based on three-axis acceleration and angular velocity.

Category	Stretch	Chest enlargement	Whole body	Leg kick	Body side	Body rotation
Single hand	99.46	99.00	100.00	100.00	100.00	100.00
Single arm	99.46	98.00	100.00	97.50	100.00	97.50
Single hip	99.46	94.74	100.00	97.50	98.00	97.50
Waist	99.46	94.74	99.00	87.50	100.00	93.50
Single leg	99.46	97.37	100.00	90.00	100.00	95.00
Single foot	97.30	89.37	100.00	97.50	99.00	94.00

RETRACTED

**Table 4:** Calibration results of three-axis acceleration.

Category	+*X*	−*X*	+*Y*	−*Y*	+*Z*	−*Z*
*x*-axis	1.19	-0.96	0.03	0.01	0.02	0.01
*y*-axis	0.03	0.02	1.02	-0.97	-0.03	0.03
*z*-axis	0.02	0.02	0.01	-0.02	0.97	-0.97

## Data Availability

No data were used to support this study.
